The article "Digital Divide of the Shattered “Iron Rice Bowl”: Economic Insecurity and ICT Access in China" was published in 2021. Journal: J Healthc Eng.

# Digital Divide of the Shattered “Iron Rice Bowl”: Economic Insecurity and ICT Access in China

**DOI:** 10.1155/2021/9122021

**Published:** 2021-08-19

**Authors:** Zhuo Li, Haijie Yin, Teng Wang

**Affiliations:** ^1^School of Humanities, Social Sciences & Law, Harbin Institute of Technology, Harbin, China; ^2^e-health Institute, School of Management, Harbin Institute of Technology, Harbin, China

## Abstract

Although economic factors account for the digital divide, the effect of economic insecurity on information communication technology (ICT) access has not been determined. The market-oriented reform of Chinese state-owned enterprises in the 1990s resulted in massive layoffs, encouraging us to investigate the relationship between economic insecurity and the digital divide. We draw on data from the China Health and Retirement Longitudinal Study (CHARLS). To handle the endogeneity related to economic insecurity, we use experience in a management position and the number of siblings as instruments for economic insecurity. With the introduction of these two instrumental variables, we find a negative relationship between economic insecurity and ICT access. This study provides insight into ICT policies involving underprivileged people in developing countries.

## 1. Introduction

The digital divide refers to the gaps in the access to ICT, ability to use ICT, and outcomes of the use of ICT [1, 2]. The digital divide has drawn attention recently because ICT access has become a barrier for potential mobile health (m-health) users in developing countries, especially for the elderly who are confronted with more health management needs [3–6]. Economic insecurity is defined as unavoidable downside economic risk (e.g., unemployment and delinquent debt status), in which individuals face hardship in their financial future [7]. The relationship between individual economic insecurity and health has been explored previously. For instance, job insecurity is linked to health inequality [8], more drug prescriptions [9], and damage to mental health [10]. However, the relationship between the digital divide and economic insecurity remains unknown. Past research has concluded that economic capacity is a major determinant of the digital divide [11], but the role of economic insecurity remains unknown. Economic insecurity is characterized by suddenness and unpredictability, such as the income inequality and unemployment that emerges in the relatively short term. Given this feature of economic insecurity, it is different from economic capacity such as social economic status (SES) and the role of economic insecurity deserves more attention.

The major objective driving this research is to investigate the relationship between economic insecurity and the digital divide. Previous research has shown that economic factors (e.g., income, education, and wealth) exacerbate the digital divide, whereas social factors involving social influence and social capital facilitate the narrowing of the digital divide [12, 13]. However, it remains unknown whether unexpected layoffs affect the digital divide. We select one proxy variable (laid off) of economic insecurity in Chinese state-owned enterprises (SOEs).

The article "Digital Divide of the Shattered “Iron Rice Bowl”: Economic Insecurity and ICT Access in China" was published in 2021. Journal: J Healthc Eng.

## 2. Background

### 2.1. Economic Insecurity and Digital Divide

The digital divide is divided into three degrees: access to IT, ability to use IT, and outcomes of the use of IT [1], and economic factors are a major source of the digital divide. For individuals, economic capacity (e.g., income and wealth) has been considered a major determinant of the digital divide [11, 14]. Other economic factors such as living in rural or urban areas [15], high-income or low-income countries [16], and communities with rich or poor facilities are related to digital access [3]. Therefore, they contribute to the digital divide and account for the structural inequality in digital access.

However, the link between economic insecurity and the digital divide remains unknown. For instance, COVID-19 as a potential source of economic insecurity (e.g., lockdown policy, social distance, and unemployment) has raised concerns because of its effect on digital access [17–19]. Additionally, predicting the emergence and consequence of economic insecurity is more difficult than regular economic effects. For example, the effect of job loss (a major source of economic insecurity) differs according to workers' age and industry [20]. Moreover, family members tend to minimize expenditure and depend more on public assistance to handle job loss [21]. Therefore, assessing the effect of economic insecurity on digital access provides a further understanding of the role of economic factors in digital access. Previously, research on economic insecurity considered two perspectives: forward looking and backward looking [22]. The forward-looking perspective emphasizes that economic insecurity is related to future financial risk; for instance, involuntary layoffs reduce income in the future. By comparison, the backward-looking perspective insists on the realized financial risk (i.e., troubles related to delinquent debt). In this study, we adopt the backward-looking perspective.

### 2.2. Reform of Chinese State-Owned Enterprises (SOEs)

In Mao Zedong's era (1950s–1970s), SOEs had two defining characteristics: being a self-sufficient community and permanent employment [23, 24]. On the one hand, this self-sufficient community provided almost free welfare goods ranging from the cradle to the grave, such as medical care, transportation, and subsided housing [23]. On the other hand, the Communist Party of China (CPC) promised permanent employment opportunities to workers, which was considered a social obligation to Chinese citizens [24]. Therefore, the tradition and institution of SOE employment were known as the “iron rice bowl.”

The article "Digital Divide of the Shattered “Iron Rice Bowl”: Economic Insecurity and ICT Access in China" was published in 2021. Journal: J Healthc Eng.

With the economic reform and open-up policy proposed in Deng Xiaoping's era (1980s–1990s), the successor of Mao Zedong, the Chinese economy transitioned from a state planning pattern to a free market in the next decades. In the process of market-based reforms, SOEs were characterized by low transparency, low competitiveness, and low profitability [25]. In 1995, new labor law was passed in which worker dismissal was allowed, suggesting that permanent employment in SOEs was no longer guaranteed. From 1995 to 2001, the number of workers in SOEs decreased by 40 percent, with 34 million workers laid off [26]. Most of the workers laid off by SOEs were characterized by age and lack of skills, reducing chances of reemployment [27]. More importantly, because of the underdeveloped social safety net in that period, leaving the self-sufficient community equaled high economic insecurity.

## 3. Data and Measurement

### 3.1. Data Collection

Two datasets are used in this study: the China Health and Retirement Longitudinal Study (CHARLS 2011) and the CHARLS Life History Survey (2014). The CHARLS is a survey of middle-aged and elderly people (aged 45 and above) in China. It is based on similar surveys, such as the English Longitudinal Study of Aging (ELSA) and the Survey of Health, Aging, and Retirement in Europe (SHARE). The CHARLS (2011) covered 150 counties and 450 communities across China, involving 17708 individuals. The participants were selected via probabilities proportional to size at the neighborhood level and geographic information systems at the household level. Therefore the repetitiveness was guaranteed [28]. The CHARLS Life History Survey (2014) includes all live respondents in the CHARLS (2011) and considers work history information (e.g., job categories, unemployment, and position of jobs). Our research includes 5460 participants, with at least one nonagriculture job. Because layoffs measure economic insecurity, participants with agriculture jobs are excluded. In this study, the age distribution of the sample is 45–59 (62.49%), 60–74 (31.70%), and 75 and above (5.81%). Males constitute 51.45%, whereas females constitute 48.55% of the sample. The sample was well balanced at the demographic level.

### 3.2. Measurement

#### 3.2.1. Economic Insecurity

Following suggestions of previous studies [7, 27], we defined economic insecurity as an unavoidable downside economic risk. We use one proxy indicator to measure economic insecurity: laid off by SOEs. In this sample of the CHARLS Life History Survey (2014), SOEs equals 1 if the respondent has the experience of being laid off by a state- or collective-controlled enterprise. In SOEs, our sample shows that 10.20% of respondents were laid off (see Table 1). The distribution of SOEs ranged from 8 percent to 14 percent in previous research [27]; therefore, it is a properly selected proxy of economic insecurity.

The article "Digital Divide of the Shattered “Iron Rice Bowl”: Economic Insecurity and ICT Access in China" was published in 2021. Journal: J Healthc Eng.

#### 3.2.2. Digital Access

The digital divide has three types: access to ICT, ability to use, and outcomes of the use of ICT [1]. In this study, we focus on the access to ICT to categorize digital access to infrastructural ICT and personal ICT. Infrastructural ICT is defined as networks facilitating information transition, storage, and delivery, for instance, Internet networks and telephone networks [29, 30]. Conversely, personal ICT refers to digital devices purchased and used by the individual consumer, such as smartphones. We applied one question to measure access to ICT infrastructure, “Does your household have a broadband Internet connection?” This sample shows that 23.77% of respondents had Internet access, whereas 76.23% had no Internet connection. Personal ICT is measured with one question, “Do members of your household own the following assets?” Mobile phone is included as an option; it appears that 83.85% of respondents had mobile phone access.

#### 3.2.3. Control Variables

*(1) Health Condition*. We divide health conditions into chronic disease and infectious disease. The CHARLS (2011) provides the self-reported number of chronic and infectious diseases diagnosed by physicians. Respondents in our sample have an average of 1.324 chronic diseases and 1.005 infectious diseases.

*(2) Education*. Education is divided into four groups: illiterate (without formal education experience), primary (elementary school), medium (middle school), and high (college and above). The distribution of the education level is 16.06% (illiterate), 36.63% (primary), 43.35% (medium), and 3.96% (high).

*(3) Wealth*. Because more than half (63.19%) of the respondents lived in rural areas, it is difficult to measure income. As suggested in the previous research [31], we adopt per capita expenditure (PCE) of households rather than income.

*(4) Residence*. The type of hukou is used to identify residents in rural and urban areas. Considering the urban-rural disparity in China, we use the category of hukou to identify respondents' residence, and 64.14% of residents lived in rural areas and 35.86% in urban areas.

*(5) Living Arrangement*. Household size and living with adult children are used to measure the living arrangements of respondents. The mean household size is measured by family members living in the same household, which is 3.566, and 55.73% of respondents live with adult children (aged above 16).

*(6) Community Infrastructure*. Community infrastructure is a multidimensional construct, ranging from facilities to services available in communities [32]. To measure community infrastructure, we asked the respondents 14 questions to confirm whether the community has infrastructure, organizations, and public services. Therefore, we calculated a composite score.

*(7) Public Investment*. Public investment is measured by the general budgetary expenditure of the respondent's local government (one hundred million RMB per 10,000 people). The general budgetary expenditure involves education, social safety net and employment effort, medical and healthcare services, agriculture forestry, and water conservation. The public investment data are from the Statistical Yearbook of China's Regional Economy (2012).

The article "Digital Divide of the Shattered “Iron Rice Bowl”: Economic Insecurity and ICT Access in China" was published in 2021. Journal: J Healthc Eng.

## 4. Empirical Strategy

The endogeneity of economic insecurity may result in biased estimation of the causal link because of potential omitted variables [33], such as employment opportunities in different industries [34]. Therefore, the probit model may contain biased estimation because of omitted variables. We adopted the two-step iv-probit method via Stata 14.0 to estimate the causal effect of economic insecurity.

First, we assessed the relationship between layoff in SOEs and two instrumental variables: management experience (ME) and siblings.

(1) $$\begin{array}{c} \text{SOEs }=\;\alpha_{\text{0}}\;+\;\alpha_{1}\text{ ME }+\;\alpha_{2}\text{ siblings }+\;\alpha_{3}\text{ control }+\varepsilon_{1}, \end{array}$$

(2) $$\begin{array}{c} \text{ICT access }=\;\beta_{\text{0}}\;+\;\beta_{1}\text{ SOEs }+\;\beta_{2}\text{ control }+\;\varepsilon_{2}. \end{array}$$

### 4.1. Instrumental Variables

Because instrumental variables (IVs) are related to instrumented variables but with no direct association with the dependent variable, we use management experience (whether the respondent used to be a manager) and siblings (number of respondent's living siblings) as IVs.

*(1) Management Experience*. Employees with management experience obtain extra advantage over their peers because management positions are related to valuable information and social connections. For instance, middle managers serve as a bridge between top managers and frontline workers, ensuring the implementation of the strategic aims of enterprises [35]. Managers have more contacts with related parties, such as consumers, government officials, and technology trends than frontline workers [36]. Therefore, managers obtain more information and resources than common workers. This provides these managers an advantage over workers in unemployment. To identify respondents with management experience, we ask the respondents what their position was (e.g., team leader, section chief, and division manager) in the middle of their jobs. If the respondent selects one of these management positions, *ME* equals 1 and the respondent will be marked as having management experience.

*(2) Siblings*. The number of the respondent's living siblings was used as an instrumental variable because social networks (e.g., siblings, relatives, and friends) have been shown to facilitate job hunting and promotion. A bigger social network predicts an advantage in employment [37, 38]. For instance, weak ties (e.g., acquaintance) provide valuable information such as job opportunities. These weak ties may provide crucial information to job seekers who do not have frequent contact with job hunters. By contrast, strong ties (e.g., siblings and friends) may provide resources more than information, such as mutual obligation between relatives [39]. Job seekers can take advantage of favoritism through social contacts, which promotes higher income [40]. Similarly, social ties influence human resource management in SOEs. For instance, reciprocity and mutual loyalty between employers and managers (Guanxi) has been found to influence recruitment and promotion [41, 42]. Guanxi is mainly based on existing family ties; if a Chinese person has a relative working in SOEs, he or she may benefit from such social connections [43]. Although guanxi also plays an important role in private-owned enterprises (POEs) in China, an SOE employee may obtain more advantage from guanxi than a POE employee because SOEs provided various scarce resources before the 1990s, such as free housing, childcare, and even spousal employment [44]. Taken together, having more siblings (a bigger social network) predicts a lower probability of being laid off by an SOE. In this study, the number of siblings is measured by the respondents' self-reported number of live siblings. In our sample, respondents have 3.30 living siblings on average.

The article "Digital Divide of the Shattered “Iron Rice Bowl”: Economic Insecurity and ICT Access in China" was published in 2021. Journal: J Healthc Eng.

### 4.2. Strength of IVs

Weak IVs refer to the situation where IVs are weakly related to dependent variables via instrumented variables, resulting in a problematic estimation of coefficients [45]. Two criteria have been applied to assess the strength of IVs. The first is the F-statistic value in the first-stage regression. As suggested by [45], if the F-statistic value of the first stage is less than 10, IVs can be considered weak. The F-value is 13.14, and the first criterion is met. The second criterion is that the direction of IVs in the first-stage regression should be consistent with theoretical assumptions. As demonstrated in Table 2, ME in SOEs (*β* *=* −0.025, *p* < 0.01) predicts less unemployment opportunities; siblings in SOEs (*β* *=* −0.008, *p* < 0.01) are negatively associated with being laid off. Thus, we conclude that ME and siblings are not weak IVs. However, the F-value of the POE model is 1.34, and the relationship between siblings and POEs is not significant, indicating that the endogeneity of POEs cannot be eliminated via the IVs; the different role of IVs can be explained by the variance in features between SOEs and POEs that we mentioned above. Therefore, SOEs are a more appropriate proxy variable to measure economic insecurity.

## 5. Results

### 5.1. Economic Insecurity and Digital Divide

We assessed Internet access and mobile phone access separately; results are shown in Table 3. In models assessing Internet access, the coefficient of SOEs in the probit model (model 1-1) is −0.159 (*p* < 0.05). When the IVs are put into models, the coefficient of SOEs in model 1-2 is −3.738 (*p* < 0.01). In the models assessing mobile phone access, the coefficient of SOEs in model 2-1 is −0.185 (*p* < 0.05), and it remains significant after introducing the IVs into model 2-2 (*β* = −3.502, *p* < 0.05).

*(1) Endogeneity Assessment*. The Wald test has been recommended to assess the endogeneity of SOEs [46]. Table 3 displays the results of the Wald test. In the model assessing Internet access with the IVs (model 1-2), the chi-square of the Wald test is 9.29 (*p* *<* *0.01*), indicating that SOEs are endogenous variables when used to assess Internet access. Omitted variables may influence the estimates. In model 2-2, similar results (chi-square = 7.39, *p* < 0.01) indicate that SOEs in models assessing mobile phone access are endogenous. Taken together, without the introduction of the IVs, the estimates will be biased.

*(2) Validity of IVs*. IVs are expected to be associated with instrumented variables but not with dependent variables. In other words, the exogeneity of instrumental variables should be guaranteed. To prove that the IVs are exogenous, we applied the generalized method of moments (GMM) as suggested in the past research. As shown in Table 4, the result of Hansen's J chi-square in the second column (Internet model) is 0.677 (*p* > 0.1), indicating the null hypothesis that the overidentifying restriction in the model is valid. That is, ME and siblings as IVs are exogenous in both models 1-2 and 2-2. However, the results of Hansen's J chi-square in the third column is 15.291 (*p* < 0.001), suggesting that at least one of the IVs is related to omitted factors. When assessing the relationship between economic insecurity and mobile phone access (model 2-2), the IVs are not valid. Therefore, the endogeneity of economic insecurity cannot be eliminated by the IVs; in other words, the effect of economic insecurity on ICT access is established in infrastructural ICT but not in personal ICT.

The article "Digital Divide of the Shattered “Iron Rice Bowl”: Economic Insecurity and ICT Access in China" was published in 2021. Journal: J Healthc Eng.

### 5.2. Wealth, Health Condition, and ICT Access

As shown in Table 3, PCE is positively related to Internet access in model 1-2 (*β* = 0.134, *p* < 0.01) and to mobile phone access in model 2-2 (*β* = 0.094, *p* < 0.01), suggesting that more wealth predicts more ICT access. Similarly, education is positively related to Internet access and mobile phone access. For instance, a higher education level predicts higher Internet access in model 1-2, and a similar pattern can be observed in mobile phone access in model 2-2. Note that a high education level is significant in the Internet access model (*β* = 0.732, *p* < 0.01) but not in the mobile phone model (*β* = 0.294, *p* > 0.1). The different role of a high level of education can be accounted for by high mobile phone access in our sample and by mobile phones as personal ICT being cheaper than infrastructural ICT. Additionally, the coefficients of residence are 0.994 (*p* *<* 0.01) in model 1-2 and 0.321 (*p* *<* 0.1) in model 2-2, indicating that living in urban areas provides more advantage than living in rural areas. Because wealth, residence, and education are indicators of social structure, the empirical findings mentioned above suggest that the digital divide among older people is part of the structural disparity.

Regarding health conditions, the number of infectious diseases has no link to digital access, whereas in model 2, chronic disease is negatively related to Internet access (*β* = −0.061, *t* = −3.10, *p* < 0.01), suggesting that only chronic disease contributes to the digital divide among elderly people. This different role can be attributed to the fact that chronic disease demands continuous treatment and daily management, and the cost is relatively higher than that of an infectious disease. For instance, families with chronic patients are confronted with higher financial risks, which further broadens inequality [47], and unsound social security systems in developing countries increase the financial pressure for elderly chronic patients [48].

## 6. Discussion

The link between economic insecurity and health inequality has drawn attention in past research. Our study reveals that economic insecurity also contributes to the digital divide. Individuals with chronic disease, especially older people, face more economic insecurity challenges. These people need more m-health services than others, but the unoptimistic conditions inevitably compromise that. The economic downside increases the digital divide for unemployed people, further broadening the existing digital divide. Workers laid off by SOEs during the 1980s to 1990s have begun to age, and the challenges related to health disparity and the digital divide should raise more concern. A more targeted policy is necessary to increase the ICT access among elderly people suffering from economic insecurity, especially for those who have been laid off by SOEs.

The article "Digital Divide of the Shattered “Iron Rice Bowl”: Economic Insecurity and ICT Access in China" was published in 2021. Journal: J Healthc Eng.

First, affordable ICT services are critical for m-health technology diffusion. Despite smart elderly care having been proposed in some developing countries to handle the problems brought about by rapid aging, affordability and access should be priorities for policy making. For instance, as shown in our empirical results, age, health conditions, and social economic factors contribute to ICT access, and economic insecurity expands this gap.

Second, mobile technology is expected to play an important role. We found that the negative effect of economic insecurity is established in infrastructural ICT (Internet access) but not in personal ICT (mobile phones). In other words, the effect of economic insecurity depends on the ICT feature. Infrastructural ICT, such as broadband connection, demands more massive investment from the community and government than personal ICT. Comparatively, personal ICT is less sensitive to economic insecurity. Because communities and families are a critical context for elderly people to receive health management, m-health services in communities can be designed to provide services via affordable equipment; for instance, short messages involving suggestions from community physicians are expected to work. Sufficient ICT infrastructure investment, such as Internet connection and mobile phone networks (2.5G, 3G, and 4G), should be provided as public goods. Subsidies from NGOs and the government are expected to increase access to infrastructural ICT.

Third, the divide in ICT access deserves more attention from m-health policy makers and researchers. In developing countries, the gap in ICT access has been a major obstacle for ICT diffusion [15]. Although the digital divide involves multiple levels (access, capacity, and outcome), efforts to increase ICT access for underprivileged populations can have a profound and positive influence. For instance, research in rural areas shows that efforts to reduce the divide in ICT access can improve ICT outcomes [12, 13].

The article "Digital Divide of the Shattered “Iron Rice Bowl”: Economic Insecurity and ICT Access in China" was published in 2021. Journal: J Healthc Eng.

## Figures and Tables

**Table 1:** Summary of variables.

Variables	Mean/percentage	Std. dev.	Min	Max
ICT access				
Internet access	23.37%			
Mobile phone access	83.72%			

Economic insecurity				
SOEs	10.20%			
POEs	1.10%			

Infectious disease	1.01	0.097	0	3
Chronic disease	1.32	1.397	0	10
PCE (log)	7.10	1.715	0	12.36

Education	2.35	0.792	1	4
Illiterate	16.19%			
Primary EDU	36.94%			
Medium EDU	42.99%			
High EDU	3.88%			

Residence	0.36	0.48	0	1
Urban (1)	35.86%			
Rural (0)	64.14%			

Gender		0.50	0	1
Female (1)	48.55%			
Male (0)	51.45%			

Age	1.433	0.601	1	3
Aged 45–59	62.49%			
Aged 60–74	31.70%			
Aged above 75	5.81%			

Household size	3.57	1.60	2	14
Coresidence children	0.56	0.50	0	1
Yes (1)	55.73%			
No (0)	44.27%			

Marital	0.909	0.288	0	1
Yes (1)	90.90%			
No (0)	9.10%			

Community infrastructure	4.349	3.747	0	14
Public investment (log)	2.86	0.84	−1.10	3.73
Siblings	3.297	1.892	0	10
ME	0.447	0.497	0	1
Yes (1)	44.65%			
No (0)	55.35%			

^*∗∗∗*^*p* < 0.01, ^*∗∗*^*p* < 0.05, ^*∗*^*p* < 0.1.

**Table 2:** Results of the first stage.

Variables	SOEs	POEs
ME	−0.025^*∗∗∗*^	−0.005^*∗*^
Siblings	−0.008^*∗∗∗*^	−0.001
Infectious disease	0.013	−0.004^*∗*^
Chronic disease	0.002	−0.000
PCE (log)	−0.004^*∗*^	0.000
Primary EDU	0.005	0.003
Medium EDU	0.003	−0.001
High EDU	−0.068^*∗∗∗*^	−0.005
Residence	0.120^*∗∗∗*^	−0.006
Gender	−0.008	−0.001
Aged 60–74	−0.054^*∗∗∗*^	−0.002
Aged above 75	−0.129^*∗∗∗*^	0.002
Household size	−0.004	−0.000
Coresidence children	0.007	0.005
Marital	−0.003	−0.004
Community infrastructure	0.006^*∗∗∗*^	0.001^*∗∗∗*^
Public investment (log)	0.000	0.001
Constant	0.127^*∗∗*^	0.013
Observations	5,460	5,460
*R*-squared	0.054	0.005

^*∗∗∗*^*p* < 0.01, ^*∗∗*^*p* < 0.05, ^*∗*^*p* < 0.1.

**Table 3:** Results of IV-probit.

Variables	Model 1-1 probit	Model 1-2 two-step IV-probit	Model 2-1 probit	Model 2-2 two-step IV-probit
SOEs	−0.159^*∗∗*^	−3.738^*∗∗∗*^	−0.185^*∗∗*^	−3.502^*∗∗*^
Infectious disease	−0.178	−0.146	−0.058	−0.014
Chronic disease	−0.068^*∗∗∗*^	−0.060^*∗∗∗*^	−0.014	−0.006
PCE (log)	0.150^*∗∗∗*^	0.134^*∗∗∗*^	0.109^*∗∗∗*^	0.094^*∗∗∗*^
Primary EDU	0.242^*∗∗∗*^	0.260^*∗∗∗*^	0.315^*∗∗∗*^	0.332^*∗∗∗*^
Medium EDU	0.442^*∗∗∗*^	0.455^*∗∗∗*^	0.587^*∗∗∗*^	0.600^*∗∗∗*^
High EDU	0.979^*∗∗∗*^	0.732^*∗∗∗*^	0.526^*∗∗∗*^	0.294
Residence	0.583^*∗∗∗*^	0.994^*∗∗∗*^	−0.061	0.321^*∗*^
Gender	0.141^*∗∗∗*^	0.111^*∗∗*^	0.062	0.033
Aged 60–74	−0.329^*∗∗∗*^	−0.522^*∗∗∗*^	−0.440^*∗∗∗*^	−0.617^*∗∗∗*^
Aged above 75	−0.223^*∗∗*^	−0.669^*∗∗∗*^	−0.770^*∗∗∗*^	−1.180^*∗∗∗*^
Household size	0.024	0.009	0.094^*∗∗∗*^	0.080^*∗∗∗*^
Coresidence children	0.688^*∗∗∗*^	0.707^*∗∗∗*^	0.370^*∗∗∗*^	0.390^*∗∗∗*^
Marital	0.144^*∗*^	0.119	0.166^*∗∗*^	0.149^*∗*^
Community infrastructure	0.085^*∗∗∗*^	0.105^*∗∗∗*^	0.017^*∗∗*^	0.035^*∗∗∗*^
Public investment (log)	0.088^*∗∗∗*^	0.088^*∗∗∗*^	0.071^*∗∗∗*^	0.071^*∗∗*^
Constant	−3.421^*∗∗∗*^	−3.061^*∗∗∗*^	−0.718^*∗∗∗*^	−0.394
Wald test of exogeneity		chi2 (1) = 9.29 Prob > chi2 = 0.0023		chi2 (1) = 7.39 Prob > chi2 = 0.0065
Observations	5,460	5,460	5,460	5,460

^*∗∗∗*^*p*< 0.01, ^*∗∗*^*p*< 0.05, ^*∗*^*p* < 0.1.

The article "Digital Divide of the Shattered “Iron Rice Bowl”: Economic Insecurity and ICT Access in China" was published in 2021. Journal: J Healthc Eng.

**Table 4:** Results of GMM.

Variables	Internet	Mobile
SOEs	−0.800^*∗∗*^	−0.690^*∗∗*^
Infectious disease	−0.010	−0.010
Chronic disease	−0.000	−0.000
PCE (log)	0.024^*∗∗∗*^	0.024^*∗∗∗*^
Primary EDU	0.088^*∗∗∗*^	0.088^*∗∗∗*^
Medium EDU	0.139^*∗∗∗*^	0.139^*∗∗∗*^
High EDU	0.073^*∗∗*^	0.073^*∗∗*^
Residence	0.071^*∗*^	0.071^*∗*^
Gender	0.008	0.008
Aged 60–74	−0.137^*∗∗∗*^	−0.137^*∗∗∗*^
Aged above 75	−0.316^*∗∗∗*^	−0.316^*∗∗∗*^
Household size	0.020^*∗∗∗*^	0.020^*∗∗∗*^
Coresidence children	0.081^*∗∗∗*^	0.081^*∗∗∗*^
Marital	0.044^*∗∗*^	0.044^*∗∗*^
Community infrastructure	0.007^*∗∗∗*^	0.007^*∗∗∗*^
Public investment (log)	0.015^*∗∗*^	0.015^*∗∗*^
Constant	0.456^*∗∗∗*^	0.456^*∗∗∗*^
Observations	5460	5460
Test of overidentifying restriction	Hansen's J chi2 (1) = .677302 (*p* = 0.4105)	Hansen's J chi2 (1) = 15.2905 (*p* = 0.0001)

^*∗∗∗*^*p* < 0.01, ^*∗∗*^*p* < 0.05, ^*∗*^*p* < 0.1.

## Data Availability

The data of the China Health and Retirement Longitudinal Study (CHARLS 2011) are available at http://charls.pku.edu.cn/pages/data/2011-charls-wave1/zh-cn.html. The data of the CHARLS Life History Survey (2014) are available at http://charls.pku.edu.cn/pages/data/2014-charls-wave3/zh-cn.html. The Statistical Yearbook of China's Regional Economy (2012) is available at http://www.stats.gov.cn/tjsj/tjcbw/201303/t20130318_451532.html.

## References

[1] Hsieh J., Rai R., Keil K. (2008). Understanding digital inequality: comparing continued use behavioral models of the socio-economically advantaged and disadvantaged. *MIS Quarterly*.

[2] UN (2019). Digital economy report. https://unctad.org/en/PublicationsLibrary/der2019_en.pdf.

[3] Hong Y. A., Zhou Z., Fang Y., Shi L. (2017). The digital divide and health disparities in China: evidence from a national survey and policy implications. *Journal of Medical Internet Research*.

[4] Jin Y., Jing M., Zhang L., Song S., Ma X. (2019). Internet access and hypertension management among the elderly population: a nationally representative cross-sectional survey in China. *Journal of Medical Internet Research*.

[5] Mars M., Scott R. E. (2010). Global E-health policy: a work in progress. *Health Affairs*.

[6] Wang T., Guo X., Wu T. (2021). Social capital and digital divide: implications for mobile health policy in developing countries. *Journal of Healthcare Engineering*.

The article "Digital Divide of the Shattered “Iron Rice Bowl”: Economic Insecurity and ICT Access in China" was published in 2021. Journal: J Healthc Eng.

[7] Osberg L. S. (2015). *How Should One Measure Economic Insecurity? OECD Statistics Working Papers*.

[8] Urbanaviciute I., De Witte H., Rossier J. (2019). Perceived job insecurity and self-rated health: testing reciprocal relationships in a five-wave study. *Social Science & Medicine*.

[9] Rocco L., Crema A., Simonato L., Cestari L. (2018). The effect of job loss on pharmaceutical prescriptions. *Social Science & Medicine*.

[10] Patel P. C., Devaraj S., Hicks M. J., Wornell E. J. (2018). County-level job automation risk and health: evidence from the United States. *Social Science & Medicine*.

[11] Wilson K. R., Wallin J. S., Reiser C. (2016). Social stratification and the digital divide. *Social Science Computer Review*.

[12] Venkatesh V., Venkatesh V., Rai A., Sykes T. A., Aljafari R., University of Arkansas, Aljafari, R., & University of Arkansas (2016). Combating infant mortality in rural India: evidence from a field study of ehealth kiosk implementations. *MIS Quarterly*.

[13] Venkatesh V., Sykes T. A. (2013). Digital divide initiative success in developing countries: a longitudinal field study in a village in India. *Information Systems Research*.

[14] Selwyn N. (2004). Reconsidering political and popular understandings of the digital divide. *New Media & Society*.

[15] (2018). *ICTs, LDCs and the SDGs: Achieving Universal and Affordable Internet in the LDCs. Thematic Report. In Partnership with the United Nations Office of the High Representative for the Least Developed Countries, Landlocked Developing Countries and Small Island Developing States (UN-OHRLLS)*.

[16] Guillén M. F., Suárez S. L. (2005). Explaining the global digital divide: economic, political and sociological drivers of cross-national internet use. *Social Forces*.

[17] Lai J., Widmar N. O. (2021). Revisiting the digital divide in the COVID ‐19 era. *Applied Economic Perspectives and Policy*.

[18] Ramsetty A., Adams C. (2020). Impact of the digital divide in the age of COVID-19. *Journal of the American Medical Informatics Association*.

[19] Watts G. (2020). COVID-19 and the digital divide in the UK. *The Lancet Digital Health*.

[20] Huttunen K., Møen J., Salvanes K. G. (2011). How destructive is creative destruction? effects of job loss on job mobility, withdrawal and income. *Journal of the European Economic Association*.

[21] Yeung W. J., Hofferth S. L. (1998). Family adaptations to income and job loss in the U.S. *Journal of Family and Economic Issues*.

[22] Rohde N., Tang K. K., Rao D. S. P. (2014). Distributional characteristics of income insecurity in the U.S., Germany, and Britain. *Review of Income and Wealth*.

The article "Digital Divide of the Shattered “Iron Rice Bowl”: Economic Insecurity and ICT Access in China" was published in 2021. Journal: J Healthc Eng.

[23] Gu E. X. (1999). From permanent employment to massive lay-offs: the political economy of ’transitional unemployment’ in urban China (1993-8). *Economy and Society*.

[24] Lee H. Y. (2000). Xiagang, the Chinese style of laying off workers. *Asian Survey*.

[25] Hassard J., Morris J., Sheehan J., Yuxin X. (2010). China’s state‐owned enterprises: economic reform and organizational restructuring. *Journal of Organizational Change Management*.

[26] Giles J., Park A. F., Cai F. (2003). How has economic restructuring affected China’s urban workers?. *SSRN Electronic Journal*.

[27] Kong N., Osberg L., Zhou W. (2019). The shattered “iron rice bowl”: intergenerational effects of Chinese state-owned enterprise reform. *Journal of Health Economics*.

[28] Zhao Y., Hu Y., Smith J. P., Strauss J., Yang G. (2014). Cohort profile: the China health and retirement longitudinal study (CHARLS). *International Journal of Epidemiology*.

[29] Guislain P. (2003). *Society in Latin America: Challenges Financing the Information Society in Latin America: Challenges and New Models*.

[30] Hanafizadeh M. R., Saghaei A., Hanafizadeh P. (2009). An index for cross-country analysis of ICT infrastructure and access. *Telecommunications Policy*.

[31] Strauss J., Thomas D. (2007). Chapter 54 health over the life course. *Handbook of Development Economics*.

[32] Li L. W., Liu J., Zhang Z., Xu H. (2015). Late-life depression in Rural China: do village infrastructure and availability of community resources matter?. *International Journal of Geriatric Psychiatry*.

[33] Gathergood J. (2013). An instrumental variable approach to unemployment, psychological health and social norm effects. *Health Economics*.

[34] Lin M.-J. (2008). Does unemployment increase crime?. *Journal of Human Resources*.

[35] Floyd S. W., Wooldridge B. (1992). Middle management involvement in strategy and its association with strategic type: a research note. *Strategic Management Journal*.

[36] Guo Y., Huy Q. N., Xiao Z. (2017). How middle managers manage the political environment to achieve market goals: insights from C hina’s state‐owned enterprises. *Strategic Management Journal*.

[37] Bian Y. (1997). Bringing strong ties back in: indirect ties, network bridges, and job searches in China. *American Sociological Review*.

[38] Granovetter M. (1983). The strength of weak ties: a network theory revisited. *Sociological Theory*.

[39] Lin N. (2002). *Social Capital: A Theory of Social Structure and Action*.

[40] Bian Y., Huang X., Zhang L. (2015). Information and favoritism: the network effect on wage income in China. *Social Networks*.

The article "Digital Divide of the Shattered “Iron Rice Bowl”: Economic Insecurity and ICT Access in China" was published in 2021. Journal: J Healthc Eng.

[41] Xianbi Huang X. (2008). Guanxi networks and job searches in China’s emerging labour market: a qualitative investigation. *Work, Employment & Society*.

[42] Zhu C. J. (2004). *Human Resource Management in China: Past, Current and Future HR Practices in the Industrial Sector*.

[43] Xian H., Atkinson C., Meng-Lewis Y. (2019). Guanxi and high performance work systems in China: evidence from a state-owned enterprise. *International Journal of Human Resource Management*.

[44] Warner M. (2009). ’Making sense’ of HRM in China: setting the scene1. *International Journal of Human Resource Management*.

[45] Stock J. H., Yogo M. (2002). Testing for Weak Instruments in Linear IV Regression.

[46] Cameron A. C., Trivedi P. K. (2010). *Microeconometrics Using Stata*.

[47] Wang Z., Li X., Chen M. (2015). Catastrophic health expenditures and its inequality in elderly households with chronic disease patients in China. *International Journal for Equity in Health*.

[48] WHO (2016). *World Report on Ageing and Health*.

[49] Li Z., Yin H., Wang T. (2021). Digital divide of shattered “iron rice bowl”: economic insecurity and digital divide in China (preprint). *JMIR mHealth and uHealth*.

